The article "Enhanced Feature Extraction-based CNN Approach for Epileptic Seizure Detection from EEG Signals" was retracted in 2023. Reasons: unreliable results or conclusions; concerns about the data; concerns about the peer review; concerns about the citations.

# Enhanced Feature Extraction-based CNN Approach for Epileptic Seizure Detection from EEG Signals

**DOI:** 10.1155/2022/3491828

**Published:** 2022-03-16

**Authors:** Puja Dhar, Vijay Kumar Garg, Mohammad Anisur Rahman

**Affiliations:** ^1^Department of Computer Science and Engineering, Lovely Professional University, Phagwara, Punjab, India; ^2^Department of Electrical and Computer Engineering, North South University, Dhaka, Bashundha, Bangladesh

## Abstract

One of the most common neurological disorders is epilepsy, which disturbs the nerve cell activity in the brain, causing seizures. Electroencephalography (EEG) signals are used to detect epilepsy and are considered standard techniques to diagnose epilepsy conditions. EEG monitors and records the brain activity of epilepsy patients, and these recordings are used in the diagnosis of epilepsy. However, extracting the information from the EEG recordings manually for detecting epileptic seizures is a difficult cumbersome, error-prone, and labor-intensive task. These negative attributes of the manual process increase the demand for implementing an automated model for the seizure detection process, which can classify seizure and nonseizures from EEG signals to help in the timely identification of epilepsy. Recently, deep learning (DL) and machine learning (ML) techniques have been used in the automatic detection of epileptic seizures because of their superior classification abilities. ML and DL algorithms can accurately classify different seizure conditions from large-scale EEG data and provide appropriate results for neurologists. This work presents a feature extraction-based convolutional neural network (CNN) to sense and classify different types of epileptic seizures from EEG signals. Different features are analyzed to classify seizures via EEG signals. Simulation analysis was managed to investigate the classification performance of the hybrid CNN-RNN model in terms of different achievement metrics such as accuracy, precision, recall, f1 score, and false-positive rate. The results validate the efficacy of the CNN-RNN model for seizure detection.

## 1. Introduction

Epilepsy is the most serious and prevalent neurological disorder [1]. The number of people suffering from epilepsy has crossed 50 million [2], which is nearly 0.6–0.8% of the whole population of the globe [3]. The most common symptom of epilepsy is the occurrence of epileptic seizures, which can occur regardless of any circumstances [4].

Electrical signals are used to detect an epileptic seizure. The normal amplitudes lie between 10 and 100 *μ*V, and the seizure patient's brain signal amplitude lies between 0.5 and 1.5 mV [5]. There are different types of seizures which include partial seizures and generalized seizures. Partial Seizure is categorized into a simple-partial seizure and complex-partial seizure while the generalized seizure is categorized into a generalized convulsive seizure and generalized nonconvulsive seizure [6].

The article "Enhanced Feature Extraction-based CNN Approach for Epileptic Seizure Detection from EEG Signals" was retracted in 2023. Reasons: unreliable results or conclusions; concerns about the data; concerns about the peer review; concerns about the citations.

Epileptic patients suffer from these highly impulsive seizures, which often cause severe damage to the nervous system, such as abnormal behaviors, loss of memory, and hypersensitivity. The electroencephalography (EEG) technique is extensively used to identify epileptic seizures from EEG recordings. Analysis of EEG signals is very important in diagnosing neurological disorders such as epilepsy. EEG monitors record the neural activities of the human brain in the form of electric signals. The EEG analyzes the electrical activities of the brain and generates patterns to classify the electrical activities as normal or abnormal. In general, EEG records brain wave patterns, and the signals are collected using an implanted device such as electrodes, which are positioned on the scalp. The collected signals are analyzed by the researchers to detect seizures from EEG signals and to record disease-related information such as type of seizure and frequency of occurrence. However, manual analysis of EEG signals is a highly complicated and intensive task since it takes many hours for neurologists to examine the recordings of EEG signals from a single patient [7, 8]. To overcome the drawbacks of the conventional process, various researchers have suggested implementing automated methods for detecting epileptic seizures. One of the major complexities associated with seizure classification is the varying morphology of seizures, which makes them difficult for neurologists to identify manually. Previous techniques focus on recognizing different patterns of neural activities that appear in EEG recordings. However, these techniques do not provide accurate results if the brain patterns are complex and unexpected. Additionally, techniques that are used for dimensionality reduction, filtration, and feature selection, cannot handle more design attributes and cannot discriminate against new patterns. These limitations often reduce their performance. Recently, deep learning (DL) and machine learning (ML) techniques have been used to overcome the limitations of conventional techniques. ML and DL algorithms are capable of extracting relevant information for identifying and classifying epileptic seizures. Several research works have validated the potential of ML algorithms in developing patient-specific models for detecting epileptic seizures [9–13]. Previously, hand-crafted attributes were employed to characterize epileptic seizures. With the advancements in EEG techniques, various researchers have suggested the application of DL-based models for detecting seizures [14–17].

The article "Enhanced Feature Extraction-based CNN Approach for Epileptic Seizure Detection from EEG Signals" was retracted in 2023. Reasons: unreliable results or conclusions; concerns about the data; concerns about the peer review; concerns about the citations.

Among various DL models, CNNs are used prominently in classification and object detection tasks [18–21]. This is due to the ability of CNN to process complex patterns using automated preprocessing, feature extraction, and dimensionality reduction. The superior attributes of CNNs make it an excellent choice for detecting epileptic seizures and hence CNNs are incorporated in this work.

The key contributions of this work can be summarized as follows:

- This study suggests a CNN-based framework for detecting epilepsy from EEG signals
- The proposed work performs feature extraction where the temporal and frequency domain features such as LBP, EMD, FFT, and DWT are extracted for epilepsy detection
- A RNN-CNN classifier is used to recognize data sequential characteristics and classify different patterns of EEG signals to detect epilepsy

The local binary patterns (LBP) feature vector is returned as a 1-by-N vector of length N, which represents the number of features. Classification, recognition, and detection use the local texture information of LBP features.

Using empirical mode decomposition (EMD), intrinsic mode functions are extracted from the signals. It is used in finding the local minima and maxima of signals.

The fast Fourier transform (FFT) is helpful in detecting the information about frequency from the EEG signals.

A discrete wavelet transforms (DWT) is used in decomposing the signals into different sets. It is helpful in finding the evolution of time in frequency.

The paper is further organized as follows: Section 2 discusses the review of existing literary works related to seizure detection using automated learning models.  Section 3 provides a comprehensive analysis of the proposed framework, which includes the design experimental procedure, which includes different stages of feature extraction.  Section 4 details the proposed CNN architecture for classification.  Section 5 presents the results of the simulation, and Section 6 concludes the paper with prominent research observations and future scope.

## 2. Related Works

Several research works have investigated the application of different detection for categorizing EEG signals to find epileptic seizures [22–26]. Conventional techniques used for detecting epileptic seizures employ hand-crafted techniques to extract relevant information from electroencephalogram signals such as time and frequency domain-related features [27–29]. These features are further used by the classifiers to categorize different EEG signals. ML and DL-based classifiers are used predominantly to classify seizures from EEG signals because of their superior classification and prediction accuracy. These classifiers use their learning mechanisms to automate the detection process and thereby allow the automatic detection of epileptic seizures with maximum accuracy. Hamad et al.,[30] used a hybrid approach known as GWO-SVM, which is composed of grey wolf optimizer (GWO) enhanced support vector machines (SVMs) for classification. The appropriate features from EEG signals were extracted using a discrete wavelet transform (DWT) technique, and the extracted features were used to train the SVM with a radial basis function. Results showed that the SVM-GWO model can effectively detect epilepsy seizures. A similar approach was proposed by Subasi et al. [13]. They proposed a hybrid approach for optimizing SVM algorithms using two-hybrid optimization algorithms such as the genetic algorithm (GA) and the particle swarm optimization (PSO) algorithm. It is shown that the hybrid SVM model is highly effective in finding epileptic seizures from EEG signals. However, these techniques depend on manual feature extraction [31], which is one of the primary limitations of these approaches. Feature extraction is an important phase for classifying seizures from EEG signals. It enhances the accuracy of classification and detection. The present work emphasizes performing classification without involving any complex feature extraction, and the potential capacity of DL algorithms has provided a new roadmap to reduce the complexity of feature extraction. Different deep learning algorithms, such as decision tree [32], SVM [33], random forest [34, 35], and recurrent neural networks (RNN) [36], based approaches are used widely for epileptic detection. Feature extraction is essential to perform before classification since it can directly process EEG samples before feeding them into the classifier. Extraction of relevant features will simplify the process of classification and improve classification accuracy. However, some of the recent works do not perform feature extraction and the DL-based models were trained directly using EEG signals [16, 37]. While the majority of these works use time-domain signals, some of the works have also used data from the frequency domain for categorizing EEG signals. It can be inferred from the existing literary works that it is essential to extract both time and frequency domain signals for analyzing the spatial characteristics of EEG signals.

The article "Enhanced Feature Extraction-based CNN Approach for Epileptic Seizure Detection from EEG Signals" was retracted in 2023. Reasons: unreliable results or conclusions; concerns about the data; concerns about the peer review; concerns about the citations.

Epilepsy is not a disease, but a neurological disorder. Many people with epileptic seizures hide their problem, and they lead a lonely life. Authors have made efforts to suggest a new epileptic seizure detection method. CNN gives very high accuracy. Deep learning techniques have the advantage of allowing the features to be automatically deduced and optimally changed for the desired outcome.

## 3. Research Methodology

The preliminary aim of the preferred research is to detect epileptic seizures from EEG signals using a feature extraction-based technique. A hybrid RNN-CNN classifier is employed for classifying different forms of EEG signals. The RESNET50 classifier is used after the feature extraction and the performance is measured. The implementation of the proposed framework involved different steps that are discussed in the following subsections.

### 3.1. Dataset Description

The data for experimental analysis was collected from an Epileptic Seizure Recognition Dataset. The obtained data is Multivariate, Time-Series data with an overall 11500 number of instances and 179 attributes. The data consists of both Integer and Real data type attributes and is suitable for performing classification and clustering tasks. More than 10 electrode systems were used for collecting the EEG signal data. The obtained data were categorized into five sets ranging from A to *E* with each set containing 100 one-channel instances. The EEG data collected from 5 healthy people were grouped into two sets namely set A and set B. Set A consists of the data when the people were in a relaxed state and Set B consisted of the data collected from the people with their eyes open. Set C consisted of the signals collected from the hippocampal formation of the opposite hemisphere of the brain. And, the EEG data collected during seizure-free intervals were grouped into set C and set D. Set *E* contained EEG signals which were measured during the seizure activity.

### 3.2. Data Preprocessing

Data processing is a preliminary step before performing feature extraction or classification tasks. In general, the obtained input EEG signals consist of redundant data with unwanted noise and artifacts. It is essential to filter out these uncertainties in order to make the data suitable for further processing. Preprocessing will ensure that only relevant signal-related information is implanted into EEG signals. The artifacts, along with external noise (usually generated due to electrode movement), get mixed with actual EEG recordings and deteriorate the quality of EEG signals and affect the classification accuracy. In this stage, the obtained EEG signal data is transformed into a two-dimensional table format in order to simplify the analysis and provide relevant information for seizure detection. For processing the input data, different feature selection models are used. In this work, the dataset used is a preprocessed, restructured dataset and is a supervised dataset that provides the class features with possible class values.

The article "Enhanced Feature Extraction-based CNN Approach for Epileptic Seizure Detection from EEG Signals" was retracted in 2023. Reasons: unreliable results or conclusions; concerns about the data; concerns about the peer review; concerns about the citations.

### 3.3. Feature Extraction

In this stage, appropriate features from a particular part of the input signal are taken out to reduce the feature values. Generally, raw EEG signals have different signal attributes, and they differ in terms of quality and length. Besides, they also possess uncertainties due to motion artifacts and noise in the background where the EEG signals are recorded. To overcome this problem, only required features are selected using feature extraction techniques. By doing so, the data dimensionality of the EEG signal data is also reduced with the help of DL algorithms. DL-based models are used for feature extraction, where these algorithms process large-scale feature sets swiftly and reduce the computational time required for processing. Feature extraction will reduce the size of the dataset and make it suitable for grouping the data into specific categories, thus eliminating the need for additional computing resources for processing large-scale data. Different feature extraction techniques such as LBP, FFT, DWT, EMD, time domain, and frequency domain features.

#### 3.3.1. Local Binary Pattern (LBP)

The LBP method identifies the intensity level of a sample in neighborhood values. In this work, a one-dimensional LBP [38] is used to take out distinct features from EEG signals. In this work, the effectiveness of LBP is investigated for classifying seizure and non-seizure EEG signals. The computation of LBP for each EEG signal is given as follows [39]:

(1) $$\begin{array}{c} {\text{LBP}}_{\text{LHS}}\left(x\left[n\right]\right)=\overset{L-1}{\underset{k=0}{\sum }}S\left(x\left[n+k-L\right]-x\left[n\right]\right)2^{2L-1-k},\\ {\text{LBP}}_{\text{RHS}}\left(x\left[n\right]\right)=\overset{2L-1}{\underset{K=L}{\sum }}S\left(x\left[n+k+1-L\right)-x\left[n\right]\right)2^{2L-1-K},\\ \text{LBP}\left(x\left[n\right]\right){=\text{LBP}}_{\text{LHS}}\left(x\left[n\right]\right){+\text{LBP}}_{\text{RHS}}\left(x\left[n\right]\right), \end{array}$$

where *L* defines the entire number of samples, x[n] defines the sample of EEG signals for which the LBP is evaluated, and the term S is given as shown in the following equation:

(2) $$\begin{array}{c} S\left(p\right)=\left\{\begin{array}{cc} 1, & \mathrm{if}\;p\geq \text{0,}\\ 0, & \text{otherwise}. \end{array}\right. \end{array}$$

The LBP of the signal is obtained by comparing the value of the EEG signal sample with its adjacent neighbors, and thereby it records the variations in the signals. Further, histograms of the LBPs from all samples are aggregated to obtain the final representation of the signals.

The article "Enhanced Feature Extraction-based CNN Approach for Epileptic Seizure Detection from EEG Signals" was retracted in 2023. Reasons: unreliable results or conclusions; concerns about the data; concerns about the peer review; concerns about the citations.

#### 3.3.2. Fast Fourier Transform (FFT)

FFT is one of the common methods used for analyzing EEG signals in the frequency domain. FFT can analyze distinct frequencies which are difficult to identify in the time domain [40]. The relative power spectral density is analyzed using FFT coefficients and, using these, the features of EEG signals are extracted and classified to detect epileptic signals using deep learning algorithms. The filtered signals, which are free from artifacts and noise, are obtained by multiplying the FFT with a high-pass filter. The FFT technique is supported by a thresholding approach to remove low-intensity signals from the filtered signals. FFT is applied to convert an image belonging to the spatial region to the frequency domain. The FFT applied to the EEG signals segments a signal sample into two different parts, namely, real and imaginary parts, which actually represent the image in the frequency domain. The Fourier transform of a signal *f* (*i*, *j*) is defined as shown in (3) [41]:

(3) $$\begin{array}{c} F\left(k\text{,}1\right)=\sum_{i=0}^{N-1}\sum_{j=0}^{N-1}f\left(i,j\right)e^{-i2\pi },\left(\frac{ki}{N}+\frac{lj}{N}\right), \end{array}$$

where *f* (*i*, *j*) represents the signal instance in the spatial region and the exponential component defines the basis function for every point present in the domain *F* (*k*, *l*) in the Fourier region. However, in the Fourier transform the segmented samples can be retransformed using an inverse Fourier transform, i.e., IFT. The IFT of the frequency of an image in the spatial region is given as

(4) $$\begin{array}{c} F\left(\mathrm{i,j}\right)=\sum_{i=0}^{N-1}\sum_{j=0}^{N-1}F\left(k,l\right)e^{-i2\pi }\left(\frac{ki}{N}+\frac{lj}{N}\right). \end{array}$$

#### 3.3.3. Discrete Wavelet Transform

DWT [42] based feature extraction is effective for detecting epileptic seizures due to its ability to extract features considering the dynamic and impulsive nature of EEG signals. The varying window size of the DWT allows it to provide accurate frequency-related information. The main advantage of DWT is its ability to provide accurate results even for nonstationary signals. The unique attribute of the DWT compared to Fourier analysis is the temporal resolution. The DWT records all image-related information along with its location, unlike Fourier transformation. The 4 sub-bands of high-frequency (LL, LH, HL, and HH) consist of functionalities in the higher frequency range of an input image. DWT finds the difference between a low-frequency sub-band image and a denoised image. After computing the difference, interpolation is performed wherein the high-frequency sub-bands are interpolated into two individual bands.

The article "Enhanced Feature Extraction-based CNN Approach for Epileptic Seizure Detection from EEG Signals" was retracted in 2023. Reasons: unreliable results or conclusions; concerns about the data; concerns about the peer review; concerns about the citations.

This convolution operation in DWT is given as follows:

(5) $$\begin{array}{c} x\left[n\right]*h\left[n\right]=\sum_{k=-\infty }^{\infty }x\left[k\right]*h\left[n-k\right]. \end{array}$$

The convolution of operation is defined using (5). The subsampling process used after the interpolation process in DWT maintains the quality of the images and information which are not related to the process are filtered out without compromising on the resolution and image quality. This process is illustrated in (6).

(6) $$\begin{array}{c} y\left[n\right]=\sum_{k=-\infty }^{\infty }h\left[k\right]*x\left[2n-k\right]. \end{array}$$

The original signal sample *x*[*n*] is subjected to filtering using a half-band high pass filter *g*[*n*] and a low-pass filter *h*[*n*]. A major portion of the redundant signal information is filtered out during the filtering process, and only the high-frequency samples are left out in the signal, which is further subsampled by factor 2. This constitutes a fundamental component of the image decomposition process, which is given as

(7) $$\begin{array}{c} Y_{\text{high}}\left[k\right]=\sum x\left[n\right]*g\left[2k-n\right],\\ Y_{\text{low}}\left[k\right]\sum_{n}x\left[n\right]*h\left[2k-n\right]. \end{array}$$

Where *y*_high_ [*k*] and *y*_low_ [*k*] represent the outputs of the high and low-frequency filters, respectively, after the subsampling of the signals.

#### 3.3.4. Empirical Mode Decomposition (EMD)

An EMD is a multiresolution decomposition method that segments a signal sample into multiple distinct frequency components known as intrinsic mode functions (IMFs) and a residue. The segmentation process is called the sifting process. Since EMD processes do not use any basis functions, it is more appropriate for nonlinear and nonstationary data analysis [43]. A signal is decomposed into ‘r1' rows and ‘c1' columns and the function *g*1(*m*, *n*) is given as

(8) $$\begin{array}{c} g1\left(r1\text{,}c1\right)\mathrm{=f}\left(r1\text{,}c1\right)-E1\left(r1\text{,}c1\right). \end{array}$$

If the above equation satisfies the conditions of IMFs, then it is considered the first IMF, denoted as BIMF_1_ (m, n). Furthermore, the sifting process is continued till all IMFs are obtained. By aggregating all the individual BIMFs, a reconstructed signal sample is obtained.

Comparison of different extraction methods is given in Table 1 where different researchers have worked on many extraction methods and also mentioned the accuracy as per their work.

## 4. RNN-CNN Architecture for Classification

Classification is performed using the hybrid CNN-RNN network, which is designed using a convolutional stack similar to the structure of RESNET50, with some minor modifications in the layer structure. The hybrid CNN-RNN architecture consists of three components: a convolutional layer, recurrent layers, and a transcription layer. The convolutional layers follow a RESNET50 style architecture where the fully-connected layers are not included while designing the system architecture. The convolutional layer can provide better feature representations of the sample images. These features are further fed to the recurrent layers, which transform them into an output sequence of labels that classify different types of EEG signals.

The article "Enhanced Feature Extraction-based CNN Approach for Epileptic Seizure Detection from EEG Signals" was retracted in 2023. Reasons: unreliable results or conclusions; concerns about the data; concerns about the peer review; concerns about the citations.

The primary layers of the proposed hybrid architect consist of convolutional layers to integrate CNN with RNN to extract epileptic seizure-related features. The performance of the convolutional layer is further given to the layers of RNN for identifying different signal patterns [44]. In this work, the convolutional layers identify the local and spatial patterns more accurately compared to RNNs.

In addition, the convolution operation of the CNN layers allows faster operation of the RNN and hence enhances its ability to detect more unique patterns. The proposed approach uses hand-crafted features along with CNN-RNN, as shown in Figure 1, to recover the accuracy and efficiency of epileptic seizure detection from EEG signals. The proposed CNN-RNN architecture consists of three convolution layers for extracting features, with one max pooling layer for reducing the dimensions of the extracted features. A fully-connected (FC) layer transforms the extracted features into feature vectors. The RNN features are extracted using the LSTM model, which is further combined with CNN layers and hand-crafted features. Finally, the FC layers are used for classifying the data.

The description of the CNN layers are as follows:

- *Convolutional layer.* This layer convolves the contributions of vertical and horizontal inputs along with filters, computing the dot product of the weights and the input, and then adding a bias term like a signal.
- *Max pooling layer.* This layer is the second most layer in the CNN architecture, which reduces the dimension of the extracted features. It overcomes the issue of overfitting by reducing the required number of parameters and running time.
- *Fully-connected layer (FC).* The FC layer is planned in such a way that it connects the output of the previous layer. The FC layer operates at the final stages of the operation to establish a connection between the output layer using the activation functions of the previous CNN layers. They construct the desired number of outputs and generate high-level features and determine which feature has the highest correlation among others.
- *Softmax layer.* The softmax layer predicts the output based on the features obtained from the fully-connected layer. It analyses the features and determines the probability of each class. Furthermore, the output of the class that has the highest probability value will be provided as the classification result.

The article "Enhanced Feature Extraction-based CNN Approach for Epileptic Seizure Detection from EEG Signals" was retracted in 2023. Reasons: unreliable results or conclusions; concerns about the data; concerns about the peer review; concerns about the citations.

## 5. Simulation Results

The classification performance of the proposed hybrid CNN-RNN framework is analyzed in terms of various performance indicators such as accuracy, precision, recall, F1 score, and false-positive rate. The output of the hybrid classifier is constructed using the elements of the confusion matrix such as true positives (TP), true negatives (TN), false positives (FP), and false negatives (FN). TP defines the number of signals identified correctly as epileptic seizures, TN represents the sample sets that can cause false implications, FN defines the signals that are wrongly identified as epileptic seizures, and FP represents the falsely optimistic signals. The performance parameters are defined in Table 1.

The equations for determining the performance metrics are defined as

(9) $$\begin{array}{c} Accuracy=\frac{\text{TP}+\text{TN}}{\text{TP}+\text{TN}+\text{FP}+\text{FN}}. \end{array}$$

Recall for a function is determined as the ratio of the cracks identified and those that are accurately classified and is given as

(10) $$\begin{array}{c} Recall=\frac{\text{TP}}{\text{TP}+\text{FN}}. \end{array}$$

Similarly, precision defines the accuracy of positive predictions.

(11) $$\begin{array}{c} Precision=\frac{\text{TP}}{\text{TP}+\text{FP}}. \end{array}$$

The *F*1 score is also defined as the *F*-measure, which is determined as the weighted harmonic mean of its precision and recall. The *F*1 score is used for measuring the accuracy of the system, which can possess values between 1 and 0. Where 1 represents the best value and 0 represents the worst value, correspondingly, the *F*1 score is defined as

(12) $$\begin{array}{c} F1score=\frac{2*\text{Precision}*\text{Recall}}{\text{Precision}+\text{Recall}}. \end{array}$$

### 5.1. Performance Evaluation

The output signal for the five dataset samples is illustrated in the following figures:

- Dataset *A* (Healthy people with open eyes)
- Dataset *B* (Healthy people with closed eyes)
- Dataset *C* (Hippocampal formation in the opposite hemisphere of the brain)
- Dataset *D* (Epileptogenic Zone)
- Dataset *E* (Seizure Activity)

The output of different datasets from dataset *A* to dataset *E* is shown in Figures 2–6. The confusion matrix representing the performance metrics of the CNN-RNN is conveyed in Figure 7.

The article "Enhanced Feature Extraction-based CNN Approach for Epileptic Seizure Detection from EEG Signals" was retracted in 2023. Reasons: unreliable results or conclusions; concerns about the data; concerns about the peer review; concerns about the citations.

The results in terms of different performance metrics are tabulated in Table 2.

### 5.2. Comparative Analysis

The outcome of the proposed method was distinguished from the existing MultiSVM approach. The confusion matrix and parameter evaluation of MultiSVM are illustrated in Figure 8 and the results are tabulated in Table 3. Evaluation of different performance metrics is given in Table 4. The comparative results of different parameters using CNN-RNN with MutliSVM are shown in Table 5.

The outcomes in terms of different performance metrics are shown in Table 2. A graphical illustration of the comparative analysis is given in Figure 9.

The feature extraction comparison table is given as

The comparative results of the proposed CNN-RNN and MultiSVM are tabulated in Table 6 and are graphically illustrated in Figure 9.

## 6. Conclusion

This paper extends a new epileptic seizure detection approach using the feature extraction method. A hybrid CNN-RNN architecture was applied to EEG signals to classify and detect epileptic seizures. The proposed approach analyzes different patterns from EEG signals and provides accurate information to the neurologists to identify different seizure types. Different feature extraction techniques, such as LBP, FFT, DWT, and EMD, were analyzed for feature extraction. The output of the proposed approach was compared with the existing MultiSVM approach. Outcomes of the experimental analysis show that the proposed approach achieved a superior classification accuracy of 93.30% in comparison to MultiSVM, whose accuracy was found to be 67.20%. In addition, the proposed approach outperforms the existing MultiSVM approach in terms of different performance metrics. For future research, this study intends to investigate other deep learning techniques for EEG signal categorization for diagnosing epilepsy.

## Figures and Tables

**Figure 1:** The flow diagram of using feature extraction methods for performance measure.

**Figure 2:** The detection result of signals for dataset *A* of healthy people with open eyes.

**Figure 3:** The detection result of signals for dataset *B* of healthy people with closed eyes.

**Figure 4:** The detection result of signals for dataset *C* with Hippocampal formation in the opposite hemisphere of the brain.

**Figure 5:** The detection result of signals for dataset *D* with epileptogenic Zone.

**Figure 6:** Detection result of signals detecting seizures from EEG signals.

**Figure 7:** Confusion matrix of hybrid CNN-RNN classifier.

**Figure 8:** Confusion matrix of the MultiSVM classifier.

**Figure 9:** Graphical illustration of comparative analysis.

The article "Enhanced Feature Extraction-based CNN Approach for Epileptic Seizure Detection from EEG Signals" was retracted in 2023. Reasons: unreliable results or conclusions; concerns about the data; concerns about the peer review; concerns about the citations.

**Table 1:** Comparison of feature extraction methods with existing work, NG means not given.

Reference	Feature extraction method	Accuracy
Acharya et al.	Continuous wavelet transform	96%
Gupta et al.	Entropy features	94.41%
Orhan et al.	Wavelet transform	99%
Guo et al.	Genetic programming-based feature extraction	98%
Fatima et al.	Wavelet transform	99.5%
Subasi	Discrete wavelet transform	NG
Sharma et al.	Frequency domain features	96.2%
Raghu et al.	Sigmoid entropy	94.21%
M. Sharma et al.	Entropy measures	94.25%
L. Wang et al.	Multidomain features model	99.25%
Jaiswal and Banka	PCA	97%
Abdelhameed and Murugavel	Wavelet-based features	95%
Sukuriti and Mitra	Variational mode decomposition	98.7%
Diykh et al.	Graph-based machine learning technique	98%
Proposed	Discrete wavelet transforms, local binary patterns, empirical mode decomposition, and fast Fourier transform	97%

**Table 2:** Performance parameters.

Observations	Epileptic seizure	Normal
Found	Positive in all ways (TP)	Falsely optimistic (FP)
Nothing was found	Negative false (FN)	True negative (TN)

**Table 3:** Evaluation of different performance metrics.

Sl No	Parameters	CNN-RNN
1	Accuracy	93.30%
2	Precision	83.2354%
3	Recall (sensitivity)	83.25%
4	Specificity	95.8125%
5	F1 score	82.6079%
6	Error	16.75%
7	False-positive rate	4.1875

**Table 4:** Evaluation of different performance metrics.

Sl No	Parameters	MultiSVM (%)
1	Accuracy	67.20
2	Precision	76
3	Recall (sensitivity)	18
4	Specificity	79.50
5	*F*1 score	66
6	Error	82
7	False-positive rate	20.50

**Table 5:** Comparative results of CNN-RNN and MultiSVM.

Sl No	Parameters	CNN-RNN	MultiSVM (%)
1	Accuracy	93.30%	67.20
2	Precision	83.2354%	76
3	Recall (sensitivity)	83.25%	18
4	Specificity	95.8125%	79.50
5	F1 score	82.6079%	66
6	Error	16.75%	82
7	False-positive rate	4.1875	20.50

**Table 6:** Feature extraction comparison.

Feature extraction name	TYPE-A healthy people with open eyes	TYPE-B healthy people with closed eyes	TYPE-C hippocampal formation of the opposite hemisphere of the brain	TYPE-D epileptogenic zone	TYPE-E seizure activity
LBP feature	0.0127	0.0036	0.0124	0.0030	0.0111
DWT feature	−6.8581	0.6013	−5.2813	−1.5043	1.8540
FFT feature	0.3504	0.6882	0.994	2.2065	0.9804
EMD feature	−0.6968	−0.8456	2.0029	−4.1189	0.5811
MFCC	0.6431	1.0029	0.8033	1.2083	0.5161
Wavelet packet entropy	−9.92*e* + 07	−5.540*e* + 08	−9.440*e* + 08	−1.101*e* + 10	−1.1270*e* + 09
Wavelet energy entropy	8.91*e* + 02	4.040*e* + 03	6.677*e* + 03	6.1628*e* + 04	8.14573*e* + 03
Lorentz plot area	2.959	10.475	9.601	27.66665	17.702
Median frequency	2.878*e* + 02	1.662*e* + 03	2.074*e* + 03	8.244*e* + 02	8.691*e* + 02
Mean frequency	1.764*e* + 03	2.045*e* + 03	4.807*e* + 02	2.043*e* + 03	2.0465*e* + 03
Standard deviation	45.0282*e* + 02	1.53*e* + 02	1.4332*e* + 02	4.4009*e* + 02	1.59*e* + 02
RMS value	52.902*e* + 02	1.127*e* + 02	1.445*e* + 02	4.4006*e* + 02	1.598*e* + 02
Band power in delta band	9.967*e* − 10	6.506*e* − 11	6.4594*e* − 09	6.0448*e* − 10	1.0704*e* − 10
Band power in theta band	6.815*e* − 10	3.097*e* − 10	3.698*e* − 09	6.8154*e* − 09	4.61*e* − 11
Band power in alpha band	1.396*e* − 09	1.709*e* − 09	5.157*e* − 09	1.7987*e* − 08	3.2983*e* − 10
Band power in beta band	7.296*e* − 10	2.519*e* − 08	1.1467*e* − 08	3.964*e* − 07	9.027*e* − 10
Band power in gamma band	2.0474*e* − 08	1.170*e* − 07	1.800*e* − 07	1.615*e* − 06	2.859*e* − 07

The article "Enhanced Feature Extraction-based CNN Approach for Epileptic Seizure Detection from EEG Signals" was retracted in 2023. Reasons: unreliable results or conclusions; concerns about the data; concerns about the peer review; concerns about the citations.

## Data Availability

The simulation experiment data used to support the findings of this study are available with the first author.
